# An Overview of the Advances in Research on the Molecular Function and Specific Role of Circular RNA in Cardiovascular Diseases

**DOI:** 10.1155/2022/5154122

**Published:** 2022-08-18

**Authors:** Lianli Yin, Yinghua Tang, Yulin Yuan

**Affiliations:** ^1^Department of Clinical Laboratory, Guangxi Academy of Medical Sciences, The People's Hospital of Guangxi Zhuang Autonomous Region, Nanning, 530021 Guangxi, China; ^2^Department of Clinical Laboratory, Guangxi Hospital of Traditional Chinese Medicine, The First Affiliated Hospital of Guangxi University of Chinese Medicine, Nanning, 530023 Guangxi, China

## Abstract

In recent years, the rate of residents suffering from cardiovascular disease (CVD), disability, and death has risen significantly. The latest report on CVD in China shows that it still has the highest mortality rate of all diseases in that country. Different from linear RNA, circular RNA (circRNA) is a covalently closed transcript, mainly through reverse splicing so that the 3′end and the 5′end are covalently connected to form a closed loop structure. It is structurally stable and abundant and has distinct tissue or cell specificity, and it is widely distributed in eukaryotes. Although circRNAs were discovered many years ago, researchers have only recently begun to slowly discover their extensive expression and regulatory functions in various biological processes. Studies have found that some circRNAs perform multiple functions in cells more used as RNA binding protein or microRNA sponge. In addition, accumulating evidence shows that the first change that occurs in patients with various metabolic diseases such as hypertension and cardiovascular disease is dysregulated circRNA expression. For cardiovascular and other related blood vessels, circRNA is one of the important causes of various complications. These findings contribute to a more comprehensive understanding and grasp of CVD, and the related molecular mechanisms of CVD should be further analyzed. Here, we review the new understanding of circRNAs in CVD and explain the role of these innovative biomarkers in the analysis and determination of other related cardiovascular events such as coronary heart disease. Thus, this study is aimed at providing new ideas and proposing more feasible medical research strategies based on circRNA.

## 1. Introduction

Circular RNA (circRNA) was first discovered in the 1970s [1], but it was not until recent years that it was included in the category of noncoding RNA molecules. For many years, circRNA had been considered to be an artifact of RNA splicing; however, driven by the increasingly updated RNA sequencing technology, scholars have fully confirmed that a large amount of circRNA is widely expressed in mammalian tissues; therefore, circRNA has become another research hotspot of noncoding RNA after microRNA (miRNA) and it has attracted an extensive amount of attention from domestic and foreign researchers [2, 3]. More than 30,000 types of circRNAs have been found in human tissues [4]. This particular type of RNA is produced following the splicing of pre-mRNA (pre-mRNA); most are produced during back splicing of one or two exons. Since it is round and lacks a free end, circRNA cannot be degraded by exonuclease, so it shows more outstanding stability than linear RNA [5]. Although the specific role of most circRNAs has not yet been clarified, it is known that a large number of circRNA can bind to miRNA to prevent it from interacting with messenger RNA (mRNA) targets (that is, circRNA acts as a miRNA sponge). Relevant results show that circRNAs have differential expression functions and play important roles in many types of diseases, including neurological diseases, cancer, cardiovascular diseases (CVDs), and immune system diseases [5–9]. In 2017, the research conclusions on the function of circRNAs show that the functions of neuron-specific circRNAs are mainly reflected in the regulation of brain sensorimotor gating and transmission synapses and then providing reliable evidence for the biological function of circRNA [10]. This article reviews the biogenesis of circRNA, its different functions, and the current understanding of circRNA in cardiac pathology.

## 2. The General Characteristics and Biological Functions of circRNA

### 2.1. The General Characteristics of circRNA

circRNA is a heterogeneous transcript. The constituent elements can be either external or internal and can be bipartite. In addition, regardless of size, there can be <100 nuclei and there can be thousands of bases, so each component between the inside and outside of the reverse shearing process is deterministic. Usually, circRNAs contain 2–3 exons and their median length is often greater than 500 nucleotides, but not more than 700 nucleotides [11, 12]. With the increasing maturity of modern biological information and RNA sequencing technology, a large amount of transcription data has appeared and circRNAs have been found in many types of cells in human organs. The proportion of expressed genes in the human brain and heart that can produce circRNAs was 20% and 9%, respectively. The expressed genes of human leukocytes can produce 10% of circRNAs, while the proportion produced by fibroblasts is about 14% [11, 13]. Through the above comparisons, it was found that the expression of circRNAs in the nervous system was overall enriched. The reason for the relatively high expression in the nervous system may be caused by the passive accumulation of neuronal cells during the slow decomposition process [14], as opposed to proliferating cells, where the expression level of circRNA is diluted during cell division. Related reports found that circRNAs produced in proliferating cells, including cancer cells, are often lower than those in terminally differentiated cells [15].

The expression level of most circRNA is 5–10% of its linear transcript; however, most circRNAs have higher expression levels relative to their linear counterparts [16]. Generally, the expression level might be low because reverse splicing is not as effective as standard splicing. Although not efficient, due to their resistance to exonuclease, some circRNAs accumulate continuously to high levels. It is fully shown that with the continuous development of human organs and the occurrence of certain diseases, the expression of circRNA will also change [17]. It has also been shown that the expression level of circRNA is increased in the developing heart [18, 19]. However, the reason for this increase is not clear, because it cannot be explained by the increase in the expression of its host genes. A study using cardiomyocytes derived from human-induced pluripotent stem cells showed that the expression of many circRNAs in these cells is dynamically regulated under conditions of chronic and acute stress (such as *β*-adrenergic stimulation) [20]. In addition, there are other stimulatory conditions, such as high temperature or oxidative stress, which may be the influencing factors of circRNA levels [21].

### 2.2. Mechanism of circRNA Formation

circRNA is formed by covalently connecting the 3′end and the 5′end through reverse splicing. This complex product containing multiple types of proteins often first excludes introns, then splices multiple exons, and gradually generates mature mRNA, which in turn catalyzes linear pre-mRNA. As observed in linear splicing, the necessary condition for the formation of circRNA is that there cannot be a connected splice site between the donor of the exon and the donor of the downstream exon; instead, it is connected to the upstream receptor site. This event produces one or more exon RNA molecules, whose 5′ and 3′ends are covalently closed and contain special inter-exon linkages but do not exist in linear transcripts, which are called reverse splicing junctions. The reason why the spliceosome selects certain exons for circularization has not been found. However, the two introns on opposite sides of the spliced exon must be closely connected. There are three main mechanisms that can achieve this requirement: circular lasso drive, intron pairing drive, and RNA binding protein (RBP).

### 2.3. The Biological Function of circRNA

In the past 5 years, research on circRNA has enabled researchers to understand the function of RNA more fully. The special structural characteristics of circRNA endow it with specific biological functions. Recent studies have shown that circRNAs play an important role in competing endogenous RNA or miRNA sponges. It can first bind to RBP, thereby attracting target RNA, and then bind to small nuclear RNA (smRNA), with the purpose of regulating splicing and transcription, enhancing polymerase II (Pol II) activity. It can also act as a modifier for protein scaffold and parental gene expression.

#### 2.3.1. circRNA as a miRNA Sponge

miRNAs are small noncoding RNA molecules, generally 20–25 nt in length; there are two main ways that they inhibit the expression of target proteins, namely, restricting the translation of target genes and mediating degradation [22, 23]. circRNA can act like competitive endogenous RNA (ceRNA). In doing so, it competitively binds to miRNA, reduces the inhibitory power of miRNA to its target gene production, and promotes expression of the target gene [24, 25]. Since circRNAs have single or multiple miRNA binding sites, they can absorb miRNAs like sponges and reduce their activities, thereby indirectly regulating the expression of miRNA target genes [26, 27]. Therefore, the molecular sponge action of miRNAs is one of the most important mechanisms of circRNA [28, 29]. circRNA competes with mRNA for binding to miRNA in the cytoplasm, thus affecting gene regulation.

#### 2.3.2. circRNA as an RBP Sponge

circRNAs can interact with Pol II and Argonaute (AGO) proteins, acting as protein regulators, affecting protein localization, species, and storage of RBPs. circMbl possesses a splicing factor muscleblind (MBL) binding site, which in turn regulates the formation of circMbl by binding to MBL, which is a complex protein self-regulation mechanism [30]. circ-Foxo3 can combine with the proteins, ternary complex generated by CDK2 and P21, and regulate cell cycle progression [31].

Most circRNAs are derived from RBP genes, which have conserved binding sites between these genes and their host RBPs. It can function by interacting with proteins. For example, there are conserved binding sites for MBL in circMbl and its flanking intron sequences. As a kind of RBP protein, MBL can regulate the splicing of MBL pre-mRNA. HuR is also an RBP that binds to PABPN1 mRNA and enhances its translation. circPABPN1 can create resistance to the binding of PABPN1 mRNA to HuR and reduce its translation through large-scale binding to HuR [32].

#### 2.3.3. circRNA as a Scaffold for Assembling Other Components

circRNAs can also act as dynamic protein scaffolds, which in turn facilitate the contact and assembly of proteins. In 2017, Du et al. discovered the first circRNA protein scaffold [33]. The protein scaffold is produced by circFoxo3 in the forkhead box O gene, which has an unusually significant binding affinity for various transcription factors, such as HIF-*α*, Id-1, FAK, and E2F1. As the level of circ-Foxo3 continues to rise, it will significantly inhibit the translocation of the above transcription factors. Related studies have also shown that circ-Amotl1, which can act as a protein scaffold, can combine with AKT and PDK1 to generate a ternary complex, which significantly promotes the nuclear translocation of pAKT [34].

#### 2.3.4. Enhanced Splicing and Transcription

Most circRNAs are stored in the cytoplasm and can be used as protein scaffolds or protein sponges, or miRNA sponges. But, combined with the related research conclusions of Li et al. on the transcriptional function of circRNAs, it was shown that some ciRNAs and EIciRNAs such as circEIF3J and circPAIP2 exist in the nucleus and interact with U1 small ribonucleoprotein (snRNP) to enhance the Pol in the RNA parent gene II transcriptional activity [35]. However, the underlying mechanism of EIciRNA is still unclear.

#### 2.3.5. Translation of circRNA

Considering the sequence of a circRNA as an internal ribosome and entry site (IRES) is a feasible route to achieve its translation; this approach allows the ribosome or initiation factor to directly bind to the translatable circRNA [36]. circRNAs can exert their biological functions through various pathways, such as regulating gene transcription, acting as a miRNA sponge, and regulating protein translation and expression; moreover, they have important regulatory effects on CVDs, including atherosclerosis (AS), myocardial infarction (MI), myocardial ischemia-reperfusion injury.

The condition for circRNA molecules to be translated into proteins or peptides is that they contain binding sites of prokaryotic ribosomes or IRES elements [37]. In recent years, it has been reported that most of the circZNF609 in the second exon produced by the human host ZNF gene adopts a splicing-dependent translation mode, and it is believed that N6-methyladenosine (m6A) can promote or enhance the translation of circRNAs [38].

## 3. The Relationship between circRNA and CVD

As the characteristics and biological functions of circRNAs have been revealed, the mechanisms of circRNAs in cardiovascular diseases have also been reported one after another and their unique mechanisms in CVD were shown in Table 1 and Figure 1.

### 3.1. Coronary Heart Disease (CHD)

CHD is one of the most fatal cardiovascular diseases. But, it is difficult to make an early clinical diagnosis of CHD [39]. The current common diagnostic methods include emergency electrocardiogram (ECG), an electrocardiogram stepping test (TET), electrical measurements, and scans (CTA) with Holter and coronary computed tomography, as well as other noninvasive examinations and invasive coronary angiography (CAG).

Not every method is perfect and has pros and cons. The disadvantage of ECG is the lack of sensitivity and specificity, the disadvantage of CTA is that the cost is too high, and the patient acceptance of CAG is too low. The circular structure of circRNA is too special to be effectively decomposed by enzymes; it is believed that circRNA can be used to diagnose coronary heart disease. Lin et al. constructed and comprehensively analyzed the competitive endogenous RNA network disorder related to circRNA in CHD; they found that circRNA may be a prospective clinical marker of CHD [40]. By analyzing the microarray of circRNAs in the peripheral blood of patients with coronary artery disease, 24 circRNAs with different expression were found, 18 were upregulated, and 6 were downregulated. Analyzed with the help of bioinformatics, the authors found that 9 kinds of circRNAs may bind to has-mir-130a-3p, leading to increased expression of TRMP3 [41]. Zhao et al. [42] screened circRNAs with different expression from patients with coronary heart disease by means of microarray analysis and finally screened out 22 circRNAs, of which 12 were upregulated and 10 were downregulated; they found that among the 22 dysregulated circRNAs, hsa_circ_0124644 had high sensitivity and specificity in the peripheral blood of patients, suggesting that hsa_circ_0124644 may have potential value as a diagnostic marker for CAD.

Moreover, studies have found that the circRNA (MICRA) derived from exon 1 of the zinc finger protein 609 (ZNF609) gene and closely associated with AMI may be a predictor of CAD [43, 44]. In normal human umbilical vein endothelial cells (HUVEC), there is substantial expression of cZNF609. Under conditions such as high glucose or hypoxia, the expression of cZNF609 in endothelial cells (ECs) in vitro and in vivo was upregulated. Conclusion found that the low expression of cZNF609 can reduce the loss of retinal vessels and inhibit pathological angiogenesis; the formation of more EC migration and tubes can also protect ECs from oxidation or hypoxia in vitro. In addition, studies have pointed out that cZNF609 can also act as a sponge for miR-150-5p, leading to enhanced expression of AKT3 (Figure 1(a)) [45]. cZNF609 can also act as a sponge for endogenous miR-615-5p, thereby inhibiting or isolating the activity of miR-615-5p, leading to increased MEF2A expression [46].

### 3.2. Atherosclerosis

AS is a chronic disease caused by a certain inflammation; it is also a pathogenic factor of coronary heart disease and ischemic stroke. Its mechanism is complex and related to many factors, including the environment, smoking, obesity, and hyperlipidemia. Genetic factors have also been confirmed to be related to AS [47]. The early stage of AS lesions is endothelial dysfunction in the arterial vascular system; it is formed by the accumulation of excess lipids in the subendothelial layer of the arterial wall; it is characterized by activated T cells and inflammatory infiltration of dendritic cells and macrophages [48]. Advanced AS often manifests as unstable atherosclerotic plaques and the formation of secondary thrombosis. Unstable atherosclerotic plaques are characterized by thin fibrous caps, vascular microcalcifications, large necrotic nuclei, and fragile new microvessels within the plaques. These pathological changes lead to lumen occlusion or rupture and hemorrhage of the vessel wall and serious consequences, such as MI and cerebral apoplexy [49, 50]. circANRIL has been reported to reduce ribosome production by vascular smooth muscle cells (VSMCs) and macrophages and reduce the continuous increase of smooth muscle cells and macrophages derived from human-induced pluripotent stem cells by combining with PES1, an important ribosomal component; thus, it plays a protective role in AS. It can be regarded as a potential target for the treatment of AS [51, 52]. miR-221, a gene that is characterized as abundant but conserved, has been reported to decrease with rupture of carotid plaques [53]. However, its role in carotid plaque rupture has not been found. Studies have shown that circR-284 adsorbs mir-221 to inhibit its activity and participates in the rupture of carotid plaques [54]. The highly conserved circLrp6 has multiple binding sites for miR-145; it can interact with multiple targets such as ITGb8, Lox, KLF4, and FASCINYes1 (Figure 1(b)). Silencing of circLrp6 prevents carotid intimal hyperplasia in mice [55]. Some studies have confirmed that there are different expressed circRNAs in human umbilical vein endothelial cells under hypoxic stress conditions, and the data show that the most expressed circRNA under this condition is cZNF292. As reported in [56], silencing of cZNF292 significantly inhibited the germination of renal tubular cells and spheroids and reduced endothelial cell proliferation. It was concluded that cZNF292 could accelerate the formation of renal tubular cells and promote endothelial proliferation under hypoxic stress conditions. Yang et al. [57] reported that circCHFR was abnormally overexpressed in low-density lipoprotein- (ox-LDL-) induced VSMCs. Through in-depth analysis, it was concluded that silencing CHFR via the miR-370/FOXO1 axis not only reduced the proliferation rate of VSMCs but also inhibited their migration (Figure 1(b)).

### 3.3. Ischemia/Reperfusion (I/R) Injury and Myocardial Infarction (MI)

Under ischemic conditions, hypoxic injury to oxygen-dependent tissues is inevitable, thereby inhibiting mitochondrial ATP production via oxidative phosphorylation. The gradually decreasing cellular ATP levels will cause the disturbance of ion homeostasis in cells. This alters the permeability of the cell membrane and enhances the activity of hydrolases and proteases, ultimately leading to cell apoptosis [58, 59]. Myocardial infarction caused by ischemia is more often treated by restoring the blood supply, but it will cause further organization of the injured area, leading to I/R injury. Myocardial I/R injury and MI are the main reasons for the high global morbidity and mortality from cardiovascular disease. The literature has proved that circRNA acts on I/R damage by studying the interaction between circRNA and miRNA [60, 61]. Relevant studies have found that the expression of circRNA CDR1as in cardiomyocytes and MI mice under hypoxic conditions is significantly upregulated [62]. In vivo overexpressed CDR1as added more MI regions, resulting in increased expression of the miR-7 target genes PARP and SP1 (Figure 1(c)). This study is the first to illustrate the role of circRNAs in myocardial infarction, and it is believed that CDR1as can provide a potential target for the treatment of myocardial infarction. Salgado et al. [43] studies have pointed out that the expression of circRNA MICRA, which is directly related to the disease, is significantly decreased in the peripheral blood of patients with MI, especially in patients with this low level, which can easily lead to the loss of left ventricular function during percutaneous reperfusion. It can be seen that the MICRA level can be used to predict whether the left ventricular function of MI patients is complete. Zhou et al. [63] found that circRNA ACR can reduce myocardial I/R damage by regulating the autophagy of the Pink1/FAM65B pathway (Figure 1(c)). Recently, studies have shown that mitochondrial fission and apoptosis circular RNA (MFCAR) can directly affect the expression of mitochondrial membrane-associated protein MTP18 during apoptosis [64]. Bioinformatics analysis and RNA downstream analysis show that MFCAR can adsorb miR-652-3p, thereby preventing it from binding to MTP18, thereby promoting the increased expression of MTP18 (Figure 1(c)). Huang et al. [65] showed that circ_SMG6 significantly increased EGR1 through the competitive binding between miR-138-5p, which would lead to myocardial I/R- and H/R-induced cell damage in mice. Furthermore, many other circRNAs are related to I/R damage. For example, cZNF292, cAFF1, cDENND4C, and cTHSD1 [56] are differentially expressed in hypoxic HUVECs. Under hypoxic conditions, the expression of cAFF and cZNF292 was upregulated but the opposite was true for cTHSD1. Using siRNA to knock down cZNF292 can reduce globular angiogenesis and cell proliferation, confirming the role of cZNF292 in I/R injury. In addition, the study found that the inhibition of miR-133 expression by circANXA2 can accelerate the death rate of cells in myocardial ischemia-reperfusion injury. circANXA2 is thought to be a potential target for the treatment of such injuries [66].

### 3.4. Cardiac Aging

Cellular senescence is caused by insufficient telomere length or by stress-induced DNA damage, which in turn causes cells to lose their mitotic activity. By screening and comparing circRNAs found in the heart, skin, lung, intestine, and other tissues of the elderly and mice, the expression level of circFoxo3 in elderly tissues was significantly increased and the *β*-galactosidase activity associated with aging (SA -*β*-gal) is also significantly increased. Since it is biologically believed that SA-*β*-gal means cell senescence, tissues in younger people show very little positive SA-*β*-gal activity in comparison to tissues in the elderly [21, 33]. Treatment with hydrogen peroxide can significantly promote the expression of circFoxo3 in different types of cells and enhance the activity of SA-*β*-gal, such as mouse primary cardiomyocytes and cardiac fibroblasts. siRNA specifically targeting the circFoxo3 can reduce the activity of SA-*β*-gal, indicating that circRNA has a different effect than linear RNA. Furthermore, circFoxo3 is related to senescence induced by doxorubicin (Dox). Using Dox to treat the diastole of the left ventricle in mice can significantly increase the intrasystolic diameter, reduce the left ventricular ejection fraction, and greatly reduce the left ventricular systolic blood pressure and (dp/dt). In Dox-treated mice, the continuous use of siRNA to knockout circFoxo3 can eliminate this damage. The RNA downstream assay confirmed that the mechanism of action of circFoxo3 consists of interacting antiaging proteins (such as ID1, E2F1, HIF1a, and FAK). The effects of circFoxo3 on the production of these proteins focus on compartmental localization. Overexpression of circFoxo3 increases the level of antistress proteins in the cytoplasmic components and reduces their translocation into the nucleus, thus canceling their transcriptional control of antiaging genes.

Recently, studies have shown that in HL1 cells treated with Dox, the expression of circttn105-11, circfhod3, circarhgap32, circstrn3, and QKI host genes was significantly downregulated [67]. And Qki has a significant protective effect on I/R-induced cardiomyocyte death and Dox-mediated senescence. Qki actively regulates the expression of circRNA from Ttn, Hhod3, and Strn3, thereby inhibiting Dox-mediated damage. Overexpression of circTtn105-11 using lentivirus will reduce the activity of caspase 3/7 and promotes cell survival. In contrast, knocking out circTtn105-11 will increase the sensitivity of cells to Dox and decreased protection from Qki (Figure 1(d)).

### 3.5. Cardiac Hypertrophy and Heart Failure

From a clinical point of view, heart failure is a variety of syndromes caused by abnormalities in the internal structure or function of the heart. It is the most severe stage of CVD with high mortality and poor prognosis. The expression of CDRlas was upregulated in plasma; both miR-135a and miR-135b levels were downregulated, heart failure patients have higher hmoxl levels compared to controls, and this finding was highly correlated with cardiac function [68]. Further research found that CDRlas, as a sponge of mir-135a and mir-135b, regulates the proliferation and apoptosis of human cardiomyocytes through mir-135a/hmoxl and mir-135b/hmoxl signaling axes, and participates in the occurrence and development of CHF (Figure 1(e)). Wang et al. [69] first identified the circRNA (called HRCR) related to the heart. HRCR can play the role of molecular sponge to “adsorb” mir-223, protect the heart through the mechanism of the HRCR/miR-223/ARC signaling pathway, and participate in the regulation of myocardial hypertrophy and heart failure. The study concluded that miR-223 transgenic mice will be transformed into cardiac hypertrophy and even lead to heart failure without any intervention and mice knocked out of the miR-223 gene did not develop cardiac pathological hypertrophy. Mechanistically, miR-223 can inhibit the expression of the antiapoptotic protein ARC by binding to the noncoding region of the target gene and HRCR can “adsorb” it to downregulate its function, promote increased expression of downstream antiapoptotic protein ARC, and inhibit the progression of pathological myocardial hypertrophy and heart failure (Figure 1(e)). Therefore, further research on the mechanism of action of circRNA is needed to help prevent and treat cardiac hypertrophy and heart failure.

### 3.6. Cardiac Fibrosis

The mechanism of cardiac fibrosis mainly lies in the excessive activation of cardiac fibroblasts. It leads to the deposition of a large amount of extracellular fibrin, resulting in the destruction of the cardiac structure and reduced function. The pathogenesis of myocardial fibrosis is complex; thus, it has not been fully elucidated. Gu et al. [70] established a cell model of myocardial fibrosis by stimulating cardiac fibroblasts with transforming growth factor *β*1; they used RNA sequencing technology to detect the circRNA expression profile in fibrotic cardiac fibroblasts. A total of 283 circRNAs were found to be abnormally expressed. Among them, there were 79 and 204 upregulated and downregulated circRNAs, respectively; the related circRNAs were verified by real-time PCR. Then, the authors constructed a ceRNA network based on the differentially expressed circRNAs combined with the prediction results obtained from bioinformatics. For modular discovery by analyzing ceRNA networks, three module genes were related to the signaling pathway of myocardial fibrosis, including TGF-*β*, PI3K-Akt, AMPK, MAPK, and other signaling pathways. It can be speculated that circRNA may regulate the occurrence and development of myocardial fibrosis. Ni et al. [71] found that the expression of circHIPK3 was significantly increased in myocardial fibroblasts and cardiac tissue after angiotensin II induction, and the proliferation and migration of myocardial fibroblasts were effectively inhibited after interfering with the expression of circHIPK3 in vitro. At the same time, after silencing it in vivo, the cardiac function and myocardial fibrosis of mice were significantly improved. To achieve this function, circHIPK3 first requires miR-29b-3p to be sponged and then to increase the expression of COL3A1, *α*-SMA, and COL1A1 (Figure 1(f)). Similarly, in a study on the myocardial tissue of diabetic mice, Zhou and Yu [72] focused on the relationship between circRNAs and myocardial fibrosis. Finally, it was found that circRNA-010567 could directly bind and reversely regulate miR-141. miR-141 can target and inhibit the formation of fibrin type I collagen, type II collagen, and α-smooth muscle actin (*α*-SMA) mediated by transforming growth factor *β*1 (TGF-*β*1). Therefore, circRNA-010567 can act on the expression of type I and type II collagen and *α*-SMA through the miR-141/TGF-*β*1 pathway, thus promoting myocardial fibrosis (Figure 1(f)).

### 3.7. Influence of the Vascular Inflammatory Response

The vascular inflammatory response can activate AS, nuclear factor *κ*B (NF-*κ*B) can initiate inflammatory response pathways, and circSirt1 can bind to tumor necrosis factor-*α* (TNF-*α*); miR-132/212 in the cytoplasm and nucleus inhibit NF-*κ*B activation, reduce the inflammatory response phenotype switch VSCMs, and inhibit the formation of neointima in blood vessels (Figure 1(g)) [73]. That study found that when ox-LDL induces an inflammatory response, circ-RELL1 can transmit positive feedback to NF-*κ*B through the miR-6873-3p/MyD88 axis to mediate the adhesion and migration of monocyte-macrophages and aggravate the inflammatory response of endothelial cells and the severity of AS [74]. Inhibiting the expression of Hsa_circ_0068087 in endothelial cells in a high-glucose environment can block the inflammatory response signaling pathway of the Toll-like receptor (TLR4)/NF-*κ*B/NOD-like receptor family protein (NLRP3), reduce endothelial cell inflammation, and induce angiogenesis and differentiation of blood vessels (Figure 1(g)) [75]. Using miRanda software, He et al. [76] predicted that Hsa_circ_0105015 and miR-637 have binding sites and the two are negatively correlated. After binding, they mediate the abnormal release and expression of inflammatory mediators and aggravate the process of oxidative stress in endothelial cells.

## 4. Limitations and Future Perspectives

Since the research on circRNAs is relatively new, most of the related studies have formed correlation or descriptive information but have not formed accurate causal judgments. With the extensive increase in RNA research, the role of circRNA has gradually become prominent. We have reason to believe that circRNA will surpass linear RNA molecules and become the next-generation “miRNA sponge.” The identification and functional study of circRNA molecules have provided new research directions for the pathogenesis and treatment of many common diseases, such as heart diseases, tumors, atherosclerosis, diabetes, and nervous system disorders. These new directions include exploring the mechanism of circRNA in the occurrence of diseases, the diagnostic value of circRNA as a molecular marker, and its role in disease treatment. Although few studies have investigated circRNA in relation to diseases, existing clinical data have found that circRNA exhibits varying degrees of expression level changes in many diseases and it affects related signal pathways or protein levels, suggesting that circRNA may be related to the disease and may be used as a potential molecular marker for disease screening and targeted therapy. We believe that further research on circRNA will create more opportunities for studies investigating the association between genes and diseases in the postgenomic era.

A significant amount of time and material costs is needed to explore the relationship between circRNA and disease through biological experiments and to study the functional role of circRNA. Some researchers have included the discovered or experimentally proven associations between circRNAs and diseases and have used them to construct a circRNA-disease association database. Due to the large amount of circRNA-related data constructed [77–80], some researchers have built computational models to predict the genetic basis of the relationship between circRNAs or miRNAs and diseases using network-based methods, machine learning, and deep learning [22, 81–83]. Prediction models based on machine learning algorithms are advantageous because the large-scale potential associations between circRNAs or miRNAs and diseases can be predicted in a short period of time. Thus, in addition to reducing the research costs and shortening the time needed to conduct the experiments, prediction models can enable biologists to specify the research scope of their study and then verify the accuracy of the predicted circRNAs/miRNAs and disease associations through biological experiments. Predicting potential circRNA/miRNA disease associations using computational methods may become a new research direction in the future, and advances in noncoding RNA association prediction research will provide valuable insights into CVD-related genetic markers and circRNAs.

In conclusion, CVD is still a major disease threatening human health and early diagnosis and intervention can significantly improve the long-term prognosis of patients and improve the quality of life. With the development of modern molecular biology technology, it will be more comprehensive and in depth to study the mechanism of circRNAs in CVD, and then, it is very likely that circRNAs will become targets and markers for the treatment of these and other related diseases.

## Figures and Tables

**Figure 1:** The mechanism of circRNA in cardiovascular disease. (a) The cZNF609 can act as a sponge for miR-150-5p, leading to enhanced expression of AKT3. (b) Mechanism of action of circRNA in atherosclerosis (the highly conserved circLrp6 has multiple binding sites for miR-145, which interacts with multiple targets, such as ITGb8, fasin, KLF4, Yes1, and lox; silencing CHFR through the miR-370/FOXO1 axis inhibits the proliferation and migration ability of VSMCs). (c) The overexpression of CDR1as in vivo promoted the increase of the MI area and enhanced the expression of the miR-7 target genes PARP and SP1; circRNA ACR can reduce myocardial I/R injury by regulating the autophagy of the Pink1/FAM65B pathway; MFCAR can adsorb miR-652-3p to prevent it from binding to MTP18, thereby increasing MTP18 expression. (d) Expression level of circfoxo3 in tissues of the elderly and its relationship with aging *β*-galactosidase activity (SA-*β*-Gal) increased significantly; knockout of circtn105-11 will increase the sensitivity of cells to Dox. (e) CDRlas acts as a sponge of miR-135a and miR-135b to target and regulate hmoxl; HRCR can act as a molecular sponge to “adsorb” miR-223, increase the expression of antiapoptotic protein ARC downstream of miR-223, and inhibit pathological cardiac hypertrophy and cardiac function exhaustion. (f) circHIPK3 sponges miR-29b-3p and upregulates *α*-SMA, COL1A1, and COL3A1; circRNA_010567 can mediate the expression of collagen type I, collagen type II, and *α*-SMA through the mir-141/TGF-*β*1 pathway, thereby promoting cardiac muscle fibrosis. (g) circRNA Sirt1 can bind to tumor necrosis factor-*α* (TNF-*α*) and miR-132/212 in the cytoplasm and the nucleus to inhibit the activation of NF-*κ*B; circ-RELL1 can act on NF-*κ*B through the positive feedback of the miR-6873-3p/MyD88 axis; inhibiting the expression of Hsa_circ_0068087 can block the inflammatory response signaling pathway of TLR4/NF-*κ*B/NOD/NLRP3.

**Table 1:** Mechanisms of circRNAs related to cardiovascular disease.

Cardiovascular disease	circRNA	miRNA/regulating target	Target gene(s)	Effect	Reference
Coronary heart disease	cZNF609	miR-150-5p	AKT3	Suppresses endothelial cell migration	[45]
	cZNF609	miR-615-5p	MEF2A	Promotes cell proliferation	[46]
Atherosclerosis	circLrp6	miR-145	Yes1, KLF4	Prevents carotid intimal hyperplasia	[55]
	circCHFR	miR-370	FOXO1	Inhibited the proliferation and migration of VSMCs	[57]
Ischemia/reperfusion injury and myocardial infarction	CDR1as	miR-7	PARP and SP1	Increase of the myocardial infarction area	[62]
	circRNA ACR	Pink1	FAM65B	Attenuates autophagy and cell death	[63]
	MFCAR	miR-652-3p	MTP18	Induces cardiomyocyte apoptosis	[64]
	circ_SMG6	miR-138-5p	EGR1	Induces cardiomyocyte apoptosis	[65]
Cardiac aging	circ-Foxo3	MDM2	p53	Promotes cell apoptosis	[33]
	circTtn105-11	Caspase 3/7	Qki5	Inhibition of cardiomyocyte apoptosis	[67]
Cardiac hypertrophy and heart failure	CDRlas	miR-135a, miR-135b	hmoxl	Promotes cell apoptosis	[68]
	HRCR	miR-223	ARC	Induces apoptosis	[69]
Cardiac fibrosis	circHIPK3	miR-29b-3p	a-SMA, COL1A1, COL3A1	Attenuates cardiac fibroblasts proliferation	[71]
	circRNA_010567	mir-141/TGF-*β*1	a-SMA	Promotes the expression of fibronectin	[72]
Influence vascular inflammatory response	circRNA Sirt1	miR-132, miR-212,	Sirt1/NF-*κ*B	Inhibits blood vessel neointima formation	[73]
	circ-RELL1	miR-6873-3p	MyD88/NF-*κ*B	Inhibits blood vessel neointima formation	[74]
	Hsa_circ_0068087	TLR4/NF-*κ*B/NOD like	NLRP3	Induces angiogenesis and differentiation of blood vessel	[75]
